# MicroRNA-573 inhibits cell proliferation, migration, and invasion and is downregulated by PICSAR in cutaneous squamous cell carcinoma

**DOI:** 10.17305/bjbms.2021.6301

**Published:** 2021-12-06

**Authors:** Yanhua Wang, Shengjian Tang, L. V. Jianping

**Affiliations:** 1 Department of Aesthetic and Plastic Surgery, Weifang People’s Hospital, Weifang, Shandong, China; 2 Institute of Plastic Surgery, Weifang Medical University, Weifang, Shandong, China

**Keywords:** MicroRNA-573, long non-coding RNA PICSAR, cutaneous squamous cell carcinoma, proliferation, migration, invasion

## Abstract

The incidence of cutaneous squamous cell carcinoma (cSCC) has been increasing in recent years. Meanwhile, microRNAs have been found to play vital roles in various cancers, including cSCC. This study aimed to investigate the expression of microRNA-573 (miR-573) in cSCC, its relationship with long non-coding RNA PICSAR and analyze its biological role. The relationship between PICSAR and miR-573 was confirmed by dual-luciferase reporter assay and Pearson’s correlation coefficient analysis. The levels of PICSAR and miR-573 were measured using quantitative Real-Time polymerase chain reaction. Cell Counting Kit-8 assay was used to evaluate the cSCC cell proliferation ability. The migration and invasion abilities of cSCC cells were evaluated by Transwell assay. PICSAR expression was increased and miR-573 was decreased in tumor tissues and cSCC cell lines. PICSAR and miR-573 can bind directly, and miR-573 expression was downregulated by PICSAR in cSCC. Overexpression of miR-573 significantly inhibited the proliferation, migration, and invasion abilities of A431 and SCC13 cells. In addition, miR-573 overexpression reversed the promotion effects of PICSAR overexpression on cSCC cell proliferation, migration, and invasion abilities. In conclusion, our findings indicated that miR-573 expression was decreased in tumor tissues and cSCC cells and was downregulated by PICSAR in cSCC. Additionally, miR-573 overexpression inhibited cSCC cell proliferation, migration and invasion, and reversed the promotion effects of PICSAR overexpression on cSCC cell biological functions. Thus, miR-573 might function as a tumor suppressor and might be involved in the regulatory effects of PICSAR on tumorigenesis in cSCC.

## INTRODUCTION

Cutaneous squamous cell carcinoma (cSCC) is the second most common cancer in humans with an increasing incidence [1]. Because of the sunlight or trauma, exposure to chemical agents, chronic wounds, or papillomavirus infection, pre-neoplastic lesions arise in the skin, which cause abnormal proliferation of keratinocytes and eventually leading to cSCC [2]. Although the clinical behavior of cSCC is generally benign, it may undergo local invasion and metastasis [3]. Squamous cell carcinoma itself is a more aggressive cancer, which is prone to lymph node and distal metastasis, and once metastatic, it is difficult to treat and has a poor prognosis. Thus, although study has found that the overall survival of patients with cSCC is extremely high, patients with advanced cSCC continue to have high morbidity and mortality [4]. Thus, it is urgent to search for new diagnostic biomarkers and thereby improve the cSCC treatment outcome.

Non-coding RNAs, especially long non-coding RNAs (lncRNAs) and microRNAs (miRNAs), have been found to be closely associated with the occurrence and development of cancers [5]. LncRNAs are defined as non-coding RNAs (ncRNAs) over 200 nucleotides in length and can regulate gene expression at epigenetic, transcriptional, and posttranscriptional levels [6]. In addition, some lncRNAs have been increasingly recognized to be involved in the progression of cSCC, such as lncRNA TINCR [30993776] and lncRNA SCARNA_2_ [7]. The important role of lncRNA PICSAR in cSCC has been reported by previous studies. For example, Piipponen et al. have reported that lncRNA LINC00162 also named P38 inhibited cSCC associated lincRNA (PICSAR) may promote cSCC tumor progression by regulating ERK1/2 signaling pathway activity [8]. In addition, PICSAR could regulate the function of cSCC cells [9]. Notably, a recent study also reported that PICSAR could promote cSCC progression by regulating miR-125b/YAP1 signaling axis [10].

It is known that lncRNAs may function as competing endogenous RNAs (ceRNAs) to regulate the biological functions or expression of miRNAs. MiRNAs are small ncRNAs that can regulate gene expression by binding to the 3’ untranslated region (3’UTR) of target mRNAs to suppress target mRNA translation or promote mRNA degradation [11]. Besides, some miRNAs have been reported to be involved in the progression of cSCC, such as miR-221 [12] and miR-497 [13]. In this study, the complementary sequence of miR-573 on the sequence of PICSAR was predicted by bioinformatics. Additionally, miR-573 was found to act as a tumor suppressor gene in some tumors and can inhibit tumor progression of melanoma [14]. Thus, we speculated that miR-573 may be associated with PICSAR and may play a role in cSCC. However, the relationship between PICSAR and miR-573 has not been reported previously, and the role of miR-573 in cSCC remains unknown.

Therefore, this study attempted to analyze the expression of miR-573 in tumor tissues of cSCC patients and cSCC cells, the relationship of miR-573 and PICSAR, as well as the effects of miR-573 expression on cell proliferation, migration, and invasion of cSCC cells.

## MATERIALS AND METHODS

### Patients and sample collection

A total of 96 cSCC patients admitted to Weifang People’s Hospital from 2014 to 2019 were recruited, all of whom had not received any anti-tumor treatment before sample collection. The inclusion criteria were: (1) patients with comprehensive case data; (2) patients without other dermatological manifestations such as liver, nasopharynx, or heart or lesions; (3) patients in whom no basal cell carcinoma was found. The tumor tissues of cSCC patients were collected, and the adjacent normal tissues (1-2 cm from the edge of the tumor tissues) were also collected. All the tissues were promptly frozen with liquid nitrogen. This study was approved by the Ethics Committee of Weifang People’s Hospital and all patients have signed informed consent.

### Cell culture and transfection

Four cSCC cell lines (A431, HSC-5, SCC13, and SCL-1) and a human keratinocyte cell line (HaCaT) were all purchased from the Shanghai Cell Bank of Chinese Academy of Sciences (Shanghai, China). The cells were cultured using Dulbecco’s modified Eagle’s medium (DMEM; Gibco; Thermo Fisher Scientific, Inc.) supplemented with 10% fetal bovine serum (FBS; Gibco; Thermo Fisher Scientific, Inc.), and maintained in a 5% CO_2_ atmosphere at 37°C. The pcDNA3.1-PICSAR, pcDNA3.1, miR-573 mimic, mimic negative control (NC) were purchased from GenePharma (Shanghai, China). The above vectors were transfected into cSCC cells using Lipofectamine 3000 transfection reagent (Invitrogen, CA, USA) according to the manufacturer’s protocols. Cells were collected after transfection for 48 hours and used for the following analyses.

### RNA extraction and quantitative real-time polymerase chain reaction (qRT-PCR)

TRIzol reagent (Invitrogen; Thermo Fisher Scientific, Inc.) was used to extract total RNA, including miRNA, from tissues and cSCC cells. A NanoDrop 2000 (Thermo Fisher Scientific, Inc.) was used to evaluate the purity and concentration of the extracted RNA. The single-stranded cDNA was then synthesized from the obtained RNA using a PrimeScript RT reagent kit (Takara Bio, Inc.) according to the manufacturer’s protocols.

The expression levels of PICSAR and miR-573 were measured using qRT-PCR, which was performed using a SYBR Green PCR Master Mix kit (Invitrogen; Thermo Fisher Scientific, Inc.) and a 7300 Real-Time PCR System (Applied Biosystems; Thermo Fisher Scientific, Inc.). All of the procedures were performed according to the manufacturer’s instructions. GAPDH was used as an internal control for PICSAR, and U6 was used as an endogenous control for miR-573. The primers used for this analysis were as follows: PICSAR forward, 5′-GGTGCCTCTTCCTCAGACATCT-3′, PICSAR reverse, 5′-CAAGGAAAAGGACTGGGCTGG-3′; GAPDH forward, 5′-GAAGGTGAAGGTCGGAGTC-3′, GAPDH reverse, 5′-GAAGATGGTGATGGGATTTC-3’; miR-573 forward, 5′-GCCGAGTAGTCAATGTGTA-3′, miR-573 reverse, 5′-CTCAACTGGTGTCGTGGA-3′; U6 forward, 5′-CTCGCTTCGGCAGCACA-3′, U6 reverse, 5′-AACGCTTCACGAATTTGCGT-3′. The expression levels of PICSAR and miR-573 were calculated using the 2^–DDCt^ method [15].

### Dual-luciferase reporter assay

At first, the binding sequence details of PICSAR and miR-573 were predicted by using starBase v2.0 (http://starbase.sysu.edu.cn/) [16]. To confirm whether there was a direct interaction between PICSAR and miR-573, a luciferase reporter assay was performed. PICSAR wild-type (PICSAR-WT) and mutant type (PICSAR-MUT) sequences were cloned into the reporter vector pGL3 (Promega, Madison, WI, USA). Then the integrated vectors were respectively co-transfected with miR-573 mimic and mimic NC into cSCC cell lines A431 and SCC13 using Lipofectamine 3000 (Invitrogen, CA, USA). Relative luciferase activity was analyzed by a Dual-Luciferase Reporter assay system (Promega, Madison, WI, USA) after 48 hours of transfection at 37°C. Firefly luciferase activity was normalized to *Renilla* luciferase activity.

### CCK-8 assay

After cell transfection, the cell proliferation was analyzed using the CCK-8 assay. The stable transfected A431 and SCC13 cells were seeded into 96-well plates at a density of 5 × 10^3^ cell/well, and then cultured in a humidified incubator at 37°C. When the cells were incubated for 0, 24, 48 and 72 hours, the CCK-8 reagent was added into the cells and the cells was further incubated for 2 hours. The optical density of samples at 450 nm was measured using a micro-plate analyzer (Bio-Rad Laboratories, Inc.) to reflect cell proliferation.

### Transwell assay

Transwell chambers (Corning, Inc.) were used to evaluate the migration and invasion abilities of A431 and SCC13 cells. The chambers without pre-coated with Matrigel (Corning, Inc.) were used for the migration assay. The upper chambers with serum-free DMEM medium were seeded with A431 and SCC13 cells (cell density of 5 × 10^5^ cell/well). The lower chambers were filled with DMEM supplemented with 10% FBS. After incubation for 24 hours at 37°C, the cells remaining on the upper membrane surface were removed, the cells in the lower chambers were fixed with 4% paraformaldehyde for 15 minutes and then stained using 0.1% crystal violet for 20 minutes. The number in five randomly selected fields was counted under an inverted light microscope (Olympus Corporation) to analyze the migration ability of cells. In performing the analysis of cell invasion ability, Transwell chambers pre-coated with Matrigel were used, and the rest procedures were the same as the migration analysis method.

### Ethics approval and consent to participate

The experimental procedures were all in accordance with the guideline of the Ethics Committee of Weifang People’s Hospital and have approved by the Ethics Committee of Weifang People’s Hospital.

A signed written informed consent was obtained from each patient.

### Statistical analysis

All experiments were repeated at least three times and the data were presented as the mean ± SD. All statistical analyses were performed using SPSS 21.0 software (SPSS, Inc., Chicago, USA) and GraphPad Prism 7.0 software (Inc., Chicago, USA). The differences between groups were assessed using Student’s *t*-test, Chi-square test, or one-way ANOVA. Correlation between PICSAR levels and miR-573 levels was assessed using Pearson’s correlation coefficient. *p* < 0.05 was considered statistically significant.

## RESULTS

### Relationship between PICSAR and miR-573 in Patients with cSCC

The binding sequences between PICSAR and miR-573 was shown in Figure 1A. According to the luciferase reporter assay results (Figure 1B and C), the relative luciferase activity in PICSAR-WT group was inhibited by miR-573 overexpression (*p* < 0.05), whereas no changes were observed in luciferase activity in PICSAR-MUT group (*p* > 0.05). The results of dual-luciferase reporter assay indicated the direct binding of miR-573 to PICSAR. Then the expression levels of PICSAR and miR-573 in the tissue samples were analyzed. The expression of PICSAR was significantly increased and the expression of miR-573 was significantly decreased in tumor tissues compared with that in normal controls (Figure 1D and E, all *p* < 0.001). As presented in Figure 1F, a negative correlation was observed between PICSAR levels and miR-573 levels (r = –0.551, *p* < 0.001).

**FIGURE 1:** Relationship between PICSAR and miR-573 in patients with cutaneous squamous cell carcinoma. (A) The binding sequences between PICSAR and miR-573. (B and C) The relative luciferase activity in PICSAR-WT group was inhibited by miR-573 overexpression, whereas no changes were observed in luciferase activity in PICSAR-MUT group. The expression of PICSAR (D) and miR-573 (E) in tumor tissues and tissues of normal controls. (F) Relative level of miR-573 was negatively correlated with relative level of PICSAR (r = –0.551, *p* < 0.001). (*p < 0.05, ***p < 0.001 vs. Untreated or Normal controls).

### Association of PICSAR and miR-573 with the clinicopathological characteristics of cSCC patients

Chi-square test was used to analyze the association of PICSAR and miR-573 expression with the clinical characteristics of cSCC patients. The median expression value of PICSAR (1.9) and miR-573 (0.5) were used as the cutoff value to classify the patients into low and high PICSAR, and low and high miR-193b expression groups, respectively. The results presented in Table 1 indicated that PICSAR and miR-573 expression were all significantly correlated with the tumor size, tumor grade, and TNM stage of cSCC patients (all *p* < 0.05). Meanwhile, patients with high PICSAR levels or low miR-573 levels contained more patients with tumors larger than 5cm in diameter, poor tumor grade, and advanced TNM stages compared with the patients with low PICSAR levels or high miR-573 levels. Therefore, PICSAR and miR-573 expression might be involved in the progression of cSCC.

**TABLE 1:** Association of PICSAR and miR-573 with the clinicopathological characteristics of cSCC patients

### Expression of PICSAR and miR-573 in cSCC cell lines

The experimental results shown in Figure 2 were obtained from three biological replicates. The expression levels of PICSAR and miR-573 were detected in the four cSCC cell lines and human keratinocyte cell line HaCaT. Consistent with the results of tumor tissues, PICSAR expression level was increased (Figure 2A**)** and miR-573 expression level was decreased (Figure 2B**)** in the cSCC cell lines compared with that in HaCaT cell line (all *p* < 0.01). We selected the A431 cells and SCC13 cell lines for the subsequent experiments. In the A431 cells and SCC13 cells, the expression of PICSAR was upregulated by pcDNA3.1-PICSAR (Figure 2C, all *p* < 0.001). As shown in Figure 2D, the expression level of miR-573 was inhibited by PICSAR overexpression in the A431 cells and SCC13 cells (all *p* < 0.001), once again proving that PICSAR directly regulates miR-573.

**FIGURE 2:** Expression levels of PICSAR and miR-573 in cutaneous squamous cell carcinoma cell lines. The expression levels of PICSAR (A) and miR-573 (B) were detected in the A431, HSC-5, SCC13 and SCL-1 cell lines as well as the human keratinocyte cell line HaCaT. (C) The expression of PICSAR was upregulated by pcDNA3.1-PICSAR in A431 cells and SCC13 cells. (D) The expression level of miR-573 was inhibited by PICSAR overexpression in the A431 cells and SCC13 cells. (**p < 0.01, ***p < 0.001 vs. HaCaT or Mock).

### MiR-573 overexpression inhibits cSCC cell proliferation, migration and invasion

The expression level of miR-573 was upregulated by miR-573 mimic in A431 cells (Figure 3A, *p* < 0.001**)** and SCC13 cells (Figure 3B, *p* < 0.001**)**. The cell proliferation abilities of A431 cells (Figure 3C, all *p* < 0.05**)** and SCC13 cells (Figure 3D, all *p* < 0.05**)** were all inhibited by miR-573 overexpression. In addition, the cell migration abilities of A431 cells (Figure 3E, *p* < 0.001) and SCC13 cells (Figure 3F, *p* < 0.001) were all inhibited by miR-573 overexpression. Moreover, miR-573 overexpression suppressed the invasion of A431 cells (Figure 3G, *p* < 0.01**)** and SCC13 cells (Figure 3H, *p* < 0.01). The above results demonstrated the potential role of miR-573 as a tumor suppressor.

**FIGURE 3:** MiR-573 overexpression inhibits cutaneous squamous cell carcinoma cell proliferation, migration and invasion. The expression of miR-573 was upregulated by miR-573 mimic in A431 cells (A) and SCC13 cells (B). In A431 cells and SCC13 cells, the cell proliferation (C and D), migration (E and F) and invasion (G and H) were all inhibited by the miR-573 overexpression. (*p < 0.05, **p < 0.01, ***p < 0.001 vs. Mock).

### MiR-573 Overexpression Reverses the Effects of PICSAR on cSCC Cell Proliferation, Migration and Invasion

The expression level of miR-573 inhibited by pcDNA3.1-PICSAR was upregulated by miR-573 mimic in A431 cells (Figure 4A, all *p* < 0.001**)** and SCC13 cells (Figure 4B, all *p* < 0.001**)**. The PICSAR overexpression promoted the cell proliferation of A431 cells and SCC13 cells, which was reversed by miR-573 overexpression (Figure 4C and D, all *p* < 0.05). The PICSAR overexpression promoted the cell migration of A431 cells and SCC13 cells, which was reversed by miR-573 overexpression (Figure 4E and F, all *p* < 0.001**)**. Consistently, the miR-573 overexpression also reversed the promotion effects of PICSAR overexpression on the cell invasion of A431 cells (Figure 4G, all *p* < 0.001**)** and SCC13 cells (Figure 4H, all *p* < 0.001).

**FIGURE 4:** MiR-573 overexpression reverses the effects of PICSAR on cutaneous squamous cell carcinoma cell proliferation, migration and invasion. The miR-573 mimic reversed the inhibitory effects of PICSAR overexpression on the expression level of miR-573 in A431 cells (A) and SCC13 cells (B). The miR-573 overexpression reversed the promotion effects of PICSAR on cell proliferation (C and D), migration (E and F) and invasion (G and H) of A431 cells and SCC13 cells. (*p < 0.05, **p < 0.01, ***p < 0.001 vs. Mock; ^#^*p* < 0.05, ^###^*p* < 0.001 vs. pcDNA3.1-PICSAR).

## DISCUSSION

Accumulating evidence indicated that miRNAs play an important role in the occurrence and development of tumor, and have the function of signal transduction and regulation of gene expression in cells [17]. In addition, some studies have showed that miRNAs play oncogenic roles or suppressive roles in human tumor progression. For instance, Liang et al. showed the decreased miR-187 expression in cervical cancer tissues and cell lines, and miR-187 exerted tumor-suppressive roles in cervical cancer cells by targeting FGF9 [18]. A study by Hu et al. reported that miR-532 was overexpressed in gastric cancer tissues and cells, exerted the promotion effects on the gastric cancer cell migration and invasion and might a potential target for gastric cancer therapy [19]. Similarly, in cSCC, some miRNAs expressions have been reported to be dysregulated and play crucial roles in tumorigenesis and development in cSCC. For instance, Zhou et al. demonstrated that miR-506 expression was upregulated in both cSCC tissues and cell lines and downregulation of miR-506 expression repressed tumorigenesis in cSCC cells by targeting P65 and LAMC1 [20]. The miR-217 expression, which was upregulated in the cSCC cell lines and was found to promote cSCC cell growth, cell cycle and invasion, contributed to the development of cSCC [21]. A study reported by Wang et al. showed that decreased miR-27a expression promoted the progression of cSCC and could serve a novel therapeutic target [22]. The aforementioned studies indicated that miRNAs might be involved in the cSCC progression, and identifying the new miRNAs affect tumor progression was very important for improving cSCC treatment.

It has been known that PICSAR played important role in the progression of cSCC [8]. Moreover, PICSAR has been demonstrated to promote cSCC progression by regulating miR-125b/YAP1 signaling axis [10]. In addition, the binding sequence details of miR-573 and PICSAR were predicted by bioinformatics. Moreover, miR-573 was found to inhibit tumor progression of melanoma [14]. Therefore, we suspected that miR-573 expression might be related to the cSCC and was regulated by PICSAR. In this study, we firstly confirmed the direct binding of miR-573 to PICSAR by dual-luciferase reporter assay. Then, we found that miR-573 expression was significantly decreased and PICSAR expression was significantly increased in tumor tissues and cSCC cells. In addition, the expression of miR-573 was inhibited by PICSAR. Moreover, PICSAR and miR-573 expression were all correlated with the tumor size, tumor grade, and TNM stage of cSCC patients. MiR-573 has been also found to be related to other types of diseases. For instance, a study by Wang et al. revealed that miR-573 played a protective role in the pathological process of rheumatoid arthritis (RA), and suggested that miR-573 might be a potential target in the treatment of RA [23]. MiR-573 expression, which was found to be significantly decreased in metastatic tissues, modulated epithelial-mesenchymal transition and metastasis of prostate cancer cells [24]. A study by Danza et al. revealed that miR-573 was downregulated in BRCA 1/2-related breast cancer, and was involved in BRCA-related breast cancer angiogenesis [25]. Besides, miR-573 was also found to be regulated by other lncRNAs, such as lncRNA SNHG1 [26] and lncRNA TTN-AS1 [27]. It is believed that the mechanisms underlying the transformation of normal keratinocytes involving the dysregulation of various key genes in cancers, and lncRNAs and miRNAs have been demonstrated as important regulators of the expression of the key genes in cancers. Besides, for the potential function of PICSAR and miR-573 in normal keratinocytes, it also has great significance to indicate the relationship between cSCC development and PICSAR and miR-573. Therefore, we speculated that miR-573 might be involved in the progression of cSCC and was downregulated by PICSAR in cSCC.

This study extends our understanding of miR-573’s functional role in cSCC. The functional role of miR-573 has previously been investigated in a variety of cancers. For example, decreased miR-573 expression was observed in pancreatic cancer cell lines, which enhanced pancreatic cancer cell proliferation, migration, and invasion via targeting TSPAN1. [28]. A study by Hu et al. showed that miR-573 caused the increase of invasion, migration, and proliferation of hepatoma cells in hepatocellular carcinoma [29]. The expression of miR-573 was decreased in degenerative nucleus pulposus cells and promoted cell viability of nucleus pulposus cells [30]. The present study conducted cell experiments to investigate the functional role of miR-573 in cSCC progression. Following transfection, the expression of miR-573 was upregulated by miR-573 mimic, and PICSAR expression was upregulated by pcDNA3.1-PICSAR. The results of cell experiments indicated that miR-573 overexpression inhibited cSCC cell proliferation, migration and invasion, suggesting that miR-573 might play suppressive role in cSCC progression. In addition, the promotion effects of PICSAR on cSCC cell biological function have been found [8]. And studies have found that some miRNAs mediated the promotion effects of PICSAR on cell biological function of other disease [31,32], including cSCC [10]. This study revealed that miR-573 overexpression reversed the promotion effects of PICSAR on cSCC cell proliferation, migration, and invasion. In addition, miR-573 has been found to reverse the effects of other lncRNAs on cell biological function, such as lncRNA FLVCR1-AS1 [33] and lncRNA TTN-AS1 [27]. Therefore, miR-573 might functions as a tumor suppressor in cSCC progression and was inhibited by PICSAR in cSCC.

There were some limitations in this study. At first, the sample size was small and future studies with a large research cohort are needed. Besides, this study only discussed the potential target genes of miR-573 and did not explore the exact target of miR-573 in cSCC. We thus performed additional in silico analysis, using TargetScan databases, to identify potential key targets of miR-573. Among them, previous studies have reported that EGFR can promote the cell proliferation and survival [34], and IL8 and CLEC2A are related to cSCC [35,36]. However, whether miR-573 could regulate EGFR, IL8 and/or CLEC2A in cSCC remains unclear, and whether miR-573 could regulate the cSCC cell biological functions through targeting EGFR, IL8, and/or CLEC2A remains also uncertain. In addition, the targets of miR-573 proposed in discussion (such as TSPAN1, E2F3, and Bax) have not been confirmed in cSCC. Thus, we will assess the correlation of miR-573 with the above targets, and assess the expression of above targets in both *in vitro* cSCC models and human cSCC tissue samples in further researches.

## CONCLUSION

In conclusion, the present study indicated that the expression level of miR-573 was decreased in tumor tissues of cSCC patients and cSCC cells, and was downregulated by PICSAR in cSCC. In addition, miR-573 overexpression inhibited the cell proliferation, migration, and invasion of cSCC cells, and reversed the promotion effects of PICSAR overexpression on cSCC cell biological functions. Overall, this study reveals that miR-573 might function as a tumor suppressor and might be involved in the biological function of PICSAR in regulating the progression of cSCC. The potential PICSAR/miR-573 axis provides a novel insight into the pathogenesis of cSCC, and may help to develop the tumor therapy targets in future.
